# CRISPR/Cas9-related technologies in liver diseases: from feasibility to future diversity

**DOI:** 10.7150/ijbs.33481

**Published:** 2020-06-01

**Authors:** Tao Xu, Li Li, Yu-chen Liu, Wei Cao, Jia-si Chen, Shuang Hu, Ying Liu, Liang-yun Li, Hong Zhou, Xiao-ming Meng, Cheng Huang, Lei Zhang, Jun Li, Huan Zhou

**Affiliations:** 1 Inflammation and Immune Mediated Diseases Laboratory of Anhui Province, Anhui Institute of Innovative Drugs, School of Pharmacy, Anhui Medical University, 81 Meishan Road, Hefei 230032, Anhui Province, China.; 2 Institute for Liver Diseases of Anhui Medical University, Anhui Medical University, Hefei 230032, China.; 3 Department of Pathology and Pathophysiology, and Bone Marrow Transplantation Center of the First Affiliated Hospital, Zhejiang University School of Medicine, Hangzhou, China.; 4 Institute of Hematology, Zhejiang University & Zhejiang Engineering Laboratory for Stem Cell and Immunotherapy, Hangzhou, China.; 5 Key Laboratory of Medical Reprogramming Technology, Shenzhen Second People's Hospital, First Affiliated Hospital of Shenzhen University, Shenzhen 518039, China.; 6 Shenzhen Qianhai Icecold IT Co., Ltd. China.; 7 Hefei Institutes of Physical Science, Chinese Academy of Sciences; Anhui Province Key Laboratory of Environmental Toxicology and Pollution Control Technology, Hefei, Anhui, PR China.; 8 National Drug Clinical Trial Institution, the First Affiliated Hospital of Bengbu Medical College.; 9 Anhui Provincial Cancer Hospital, West Branch of The First Affiliated Hospital of USTC, Division of Life Sciences and Medicine, University of Science and Technology of China, Hefei, Anhui, 230031, P.R. China.

**Keywords:** CRISPR/Cas9, viral hepatitis, hepatocellular carcinoma (HCC), clinical research

## Abstract

Liver diseases are one of the leading causes of mortality in the world, mainly caused by different etiological agents, alcohol consumption, viruses, drug intoxication, and malnutrition. The maturation of gene therapy has heralded new avenues for developing effective interventions for these diseases. Derived from a remarkable microbial defense system, clustered regularly interspaced short palindromic repeats/CRISPR-associated proteins 9 system (CRISPR/Cas9 system) is driving innovative applications from basic biology to biotechnology and medicine. Recently, the mutagenic function of CRISPR/Cas9 system has been widely adopted for genome and disease research. In this review, we describe the development and applications of CRISPR/Cas9 system on liver diseases for research or translational applications, while highlighting challenges as well as future avenues for innovation.

## Introduction

Genome-editing technologies such as zinc-finger nucleases (ZFNs) and transcription activator-like effector nucleases (TALENs) have begun to enable targeted genome modifications, but they still have some restrictions 1. As far as ZFNs, Two ZFNs are needed at either side of the double-strand breaks (DSBs), increasing specificity while escalating the size of the complex hindering delivery at the same time. TALENs can almost target any DNA sequence. However, TALENs are not easy to deliver *in vivo* due to a large molecular size 2. But the situation changed with the development of clustered regularly interspaced short palindromic repeats/CRISPR-associated proteins 9 (CRISPR/Cas9) genome editing. CRISPR/Cas9 genome editing is a natural RNA-mediated adaptive defense mechanism found in some prokaryotic organisms 3. It has rapidly become the most promising genome editing tool with great potential to revolutionize biomedical treatment 4. Studies have shown that the ease of retargeting the system to modify genomic sequences greatly exceeds the capability of ZFNs and TALEs, while offering similar or greater efficiencies. Many physicians and scientists are now searching for the best clinical applications for this promising technology 5.

On the other hand, liver disease incidence is increasing year by year 6. Frequently, liver diseases are initiated by oxidative stress and inflammatory reaction which leads to the excessive production of extracellular matrix (ECM), followed by a progression to hepatitis, fibrosis, cirrhosis and hepatocellular carcinoma (HCC) 7. Additionally, steatosis can cause nonalcoholic steatohepatitis (NASH) and this is also accompanied with advanced fibrosis, cirrhosis, and ultimately HCC 8. A major milestone in the development of CRISPR/Cas9 was its adaptation for use in mammalian cells, which provided researchers with a powerful tool to study genetic perturbations in tissue homeostasis and disease 1. In this review, we sum up recent progress using this genome editing technology and explore its potential clinical applications, strategies, and challenges in the liver.

## Overview of CRISPR/Cas9 technique

The CRISPR clustered repeats were first reported by Nakata and colleagues in 1987 9. They discovered a curious set of 29 nt repeats were interspaced by five intervening 32 nt nonrepetitive sequences when studying the iap enzyme involved in isozyme conversion of alkaline phosphatase in E. coli 9. However, the significance of this discovery was not immediately recognized at the time by the scientific community. 13 years later, in 2000, this sequence was described again and was proposed to exist in prokaryotes. At that time, no such sequence has been named 10. It was not until 2002 that this novel family of repetitive DNA sequences, present among both domains of the prokaryotes (Archaea and Bacteria), but absent from eukaryotes or viruses, once again caught the attention of researchers. This family is referred as CRISPR, which is characterized by direct repeats, varying in size from 21 to 37 bp, and interspaced by similarly sized nonrepetitive sequences 11. CRISPR has since opened its legendary path. Then five years later, the role of CRISPR in prokaryotic acquired immunity was confirmed for the first time 12. Between 2007 and 2011, CRISPR/Cas9 has shown great appeal to researchers and discoveries about CRISPR are springing up. In 2010, CRISPR/Cas systems are classified into three types (I- III) based on the structure and sequence of Cas proteins (Cas3 for type I, Cas9 for type II and Cas10 for type III), with a further division into several subtypes 3,13,14. Afterward, one study proposed trans-activating crRNA (tracrRNA) forms a duplex structure with CRISPR-derived RNA (crRNA) in association with Cas9 15. Since then, CRISPR/Cas9 has entered an era of rapid development. Based on previous researches published, biochemical studies revealed that Cas9 is a programmable RNA-guided DNA endonuclease, and the Cas9-crRNA-tracrRNA complex cleaves double-stranded DNA (dsDNA) targets complementary to the 20-nucleotide guide sequence in the crRNA 16,17. In 2013, the research on CRISPR/Cas9 finally moved from prokaryote to eukaryote 5. It was reported that the CRISPR/Cas9 system can be used for genome editing in mammalian cells. The following studies found that the CRISPR/Cas9 system can be utilized to generate KO mice efficiently 18. At this point, CRISPR/Cas9 ultimately came to the world as genetic engineering technology. With the deepening of exploration, the first high throughput screening of CRISPR long-chain non-coding RNA (lncRNA) gene was completed and a pregenome RNA (pgRNA) library was constructed using lentivirus as a vector. The genome-wide screening of nearly 700 genes in the human liver cancer cell line Huh 7.5 OC associated with cancer or other diseases with lncRNA was performed 19. In October 2016, Lu you et al. launched the world's first human application of CRISPR, in which T cells were isolated from patients recruited, and CRISPR technology was used to KO the PD-1 gene in the cell 20. Another breakthrough was achieved by the Zhang F team in 2017, which fused RNA-editing enzymes into targeted RNA-targeted Cas proteins, which can artificially edit specific nucleotides in human cells. This method called RNA Editing for Programmable A-to-I replacement (REPAIR) 21. However, this technology has also caused controversy among some researchers, who believe it may be a double-edged sword. Treatment by CRISPR/Cas9 may increase the risk of cancer in patients 22,23. Based on this, in 2018, single-base editing is a further development of gene-editing technology CRISPR, which may break the cancer panic of CRISPR 24. In summary, as an important, emerging and cutting-edge gene-editing technology, CRISPR/Cas9 plays an important role in genetic engineering (**Figure 1**).

The working mechanism of the CRISPR/Cas system differs from other genome editing platforms, for it uses an RNA molecule more than a protein to recognize DNA 25. CRISPR/Cas systems are classified into three types (I-III). All these types have three essential components in common: the CRISPR array, the upstream leader sequence, and the Cas genes. The CRISPR array consists of identical repeats with a length of 23-47 bp. The CRISPR/Cas leader region acts as a promoter for the transcription of the CRISPR array. The Cas genes encode the Cas proteins, containing RuvC- and HNH-like catalytic domains, which cleave the targeted DNA. Recognition of the target sequence by the Cas proteins is facilitated by the presence of the protospacer-associated motif (PAM). This sequence is usually 2-4 nucleotides long and flanks the target site. It is absent from the endogenous loci so it can prevent CRISPR/Cas auto cleavage and add specificity to targeting 3. Types I and III CRISPR loci contain multiple Cas proteins, now known to form complexes with crRNA to facilitate the recognition and destruction of target nucleic acids. Type II CRISPR/Cas system is the simplest in terms of the number of genes for types I and III have more various cas genes 14. The type II CRISPR/Cas system is the most commonly used CRISPR/Cas system for gene editing applications, which use the Cas9 protein, the only enzyme that mediates target DNA cleavage within the Cas gene cluster, through recognizing the relevant PAM sequence 26. Therefore, the majority of CRISPR-based technology development has focused on the signature Cas9 nuclease from type II CRISPR systems 27. In type II systems, a small non-coding RNA called the tracrRNA, is partially complementary to the CRISPR repeats, forming an RNA duplex with crRNA. This RNA hybrid is recognized and processed to form mature gRNA and then is combined with Cas9. The complex, including the tracrRNA, recognizes invading DNA and inactivates it by cleavage 3. In addition to Cas9, all identified type II CRISPR-Cas loci contain Cas1 and Cas2 and most type II loci also encode a tracrRNA, which is partially complementary to the repeats within the respective CRISPR array 14. Since the establishment of a new generation of CRISPR/Cas9 gene-editing system, it has been widely believed that Cas9 nuclease cleans DNA double strands to produce flat ends. But amazingly, DNA double-strand cleavage induced by Cas9 nuclease can produce protruding terminal. This latest study has fundamentally challenged the existing understanding of DNA cleavage by Cas9 nucleases and may become a turning point discovery and original innovation in the new generation of CRISPR/Cas9 gene-editing systems 28. It lays a solid foundation for optimizing and modifying gene-editing technology (**Figure 2**).

In addition to generating frameshift-derived KO mice, the CRISPR/Cas9 system offers many other applications, such as point mutations, small insertions, large deletions, large insertions, and multiplex modification. In 2018, a significant breakthrough in gene therapy was achieve by Professor Zhang F and Professor David Liu, showing that single-base editing technology can accurately edit individual bases on DNA or RNA with a very high degree of flexibility and efficiency 24. By using this technology, we can precisely repair a series of point mutations which lead to diseases, write genetic mutations that help prevent disease or regulate the expression of disease-causing genes.

The CRISPR/Cas9 has been particularly hot in the field of liver research. For example, the CRISPR/Cas9 system was capable of disrupting the intrahepatic HBV genome, with a significant increase of hepatitis B surface antigen (HBsAg) in an HBV hydrodynamics-mouse model 29. At present, gene editing is being developed to treat a variety of chronic disorders and has exciting potential for curing liver diseases 3.

## Current applications in liver diseases

Recently, the CRISPR/Cas9 system is utilized as a precise and time- and cost-saving technique for gene KO, while liver diseases vary and suitable options for the therapy adopting CRISPR/Cas9 technique are often limited 3, 30. Treatment outcomes depend not only on patient history and disease type but also on the progression of the disease and prior treatment. Overall, gene therapy using DNA modification is now possible and available, which may be exploited to achieve long term therapeutic benefit 3 (**Figure 3**).

### Viral hepatitis

Hepatitis B virus (HBV) infection is a major global health problem, despite the availability of effective vaccines 31. Approximately 240 million people are chronically infected with HBV worldwide 32. Viral infections are major risk factors for chronic liver diseases. With carriers exhibiting increased susceptibility to cirrhosis and HCC, more than 700, 000 people die from HBV-associated diseases each year 3,31. Persistence of HBV covalently closed circular DNA (cccDNA) under current antiviral therapy is the major barrier to the eradication of chronic hepatitis B (CHB) 29. For instance, although nucleos(t)ide analogs can inhibit HBV replication efficiently, they cannot eliminate cccDNA and it persists in hepatocyte nuclei 31. Thus, HBV has emerged as an attractive target for CRISPR/Cas9 in the laboratory and curing CHB will require novel strategies for specific disruption of cccDNA 29.

Lin et al. were the first group to use CRISPR/Cas9 to target HBV 29. Additionally, multiple studies have showed antiviral gRNAs can be promoted to expression by co-injecting HBV-encoding plasmid DNA and CRISPR/Cas9 vectors through the animal's tail vein in hydrodynamics-HBV *in vivo* models, which will eliminate the virus production efficiently 33. Subsequently, Dong et al. used CRISPR/Cas9 target to establish cccDNA expression model *in vivo* 34. Moreover, DNA polymerase κ (POLK), a Y-family DNA polymerase with maximum activity in non-dividing cells, substantially contributes to cccDNA formation during de novo HBV infection. Depleting gene expression of POLK by CRISPR/Cas9 KO inhibited the conversion of relaxed circular DNA (rcDNA) into cccDNA, thereby diminishing cccDNA formation and the viral infection 35. A recent study indicated that HBV replication markers were effectively inhibited following the delivery of SaCas9 and S gene targeting gRNA into HepG2.2.15 cells 36.

HCV (hepatitis C virus) is one of the leading causes of chronic hepatitis, liver cirrhosis and HCC and infects approximately 170 million people worldwide 37. The Cas9 variant from Francisella novicida (FnCas9) is reported to be capable of binding the mRNA from HCV, and thus inhibiting HCV protein expression. Interestingly, FnCas9 is also able to target DNA for double-strand cleavage, showing the possibility for a dual-targeting strategy 38. Besides, CRISPR/Cas9 could be also used to target host factors that are essential for viral replication. These two targeting strategies may reduce the possibility of a severe liver injury for therapy trials 39 (**Table 1**).

Additional studies are needed to assess whether CRISPR/Cas9 holds the therapeutic potential to limit productive infections *in vivo* and are capable of eradicating multiple cccDNA copies present in infected hepatocytes 33. In the future, the CRISPR/Cas9 system may be the most feasible approach for targeting HBV cccDNA. It is necessary to further improve the strategy to maximize the effects and minimize toxicity 31.

### HCC

HCC is the fifth most common tumor and the third leading cause of cancer mortality worldwide 40. CRISPR/Cas9-mediated gene KO is a powerful technique for precise gene modification in numerous cell types, which provides a theoretical basis for the development of novel therapies for many cancers, including HCC.

G9a is a lysine methyltransferase and its primary function is to di-methylate lysine 9 of histone H3 (H3K9me2). G9a-dependent H3K9me2 can recruit H3K9me2-binding proteins preventing transcriptional activation, which leads to gene silencing 41. The up-regulation of G9a indicates poor prognosis in HCC 42. Experimentally, G9a-KO by using CRISPR/Cas9 can suppress the proliferation and migration of HCC cells *in vitro* and inhibited HCC tumorigenicity *in vivo*, suggesting that targeted applications of CRISPR/Cas9 system could disrupt the HCC development both *in vitro* and *in vivo* 43. Moreover, much of evidence proved that total eukaryotic elongation factor 2 (eEF2) and phosphorylated eEF2 at threonine 56 are prognostic markers for overall survival of HCC-patients and the regulating eEF2 kinase is a potential drug target for tumor therapy 44. eEF2 plays an essential role in the GTP-dependent translocation of the ribosome along mRNA 45. CRISPR/Cas9-mediated eEF2 kinase KO was performed in the HCC cell line, indicating that both the cell proliferation and the growth rate decrease with the elimination of eEF2 kinase by CRISPR/Cas9 in HCC cells 44. Nuclear receptor coactivator 5 (NCOA5) plays an important role in the development of a variety of malignancies. NCOA5-KO HCC cells (LM3) by CRISPR/Cas9-mediated genome editing has been successfully generated, finding that NCOA5-KO suppresses epithelial-mesenchymal transition (EMT) in LM3, which leads to impaired cell proliferation and migration. EMT, a complex process, plays an important role in the advance of cancer 46. Additionally, CXC chemokine receptor 4 (CXCR4) is a specific receptor of chemokine stromal cell-derived factor-1 (CXCL12). CXCL12 has a strong chemotaxis effect on lymphocytes. Numerous studies have demonstrated a marked association between high CXCR4 expression and the invasiveness, progression, and metastasis of HCC 47. Targeting CXCR4 by CRISPR/Cas9 could inhibit HepG2 cell proliferation, migration and invasion, reversed EMT, increased chemosensitivity and decrease the malignancy of HCC *in vitro* and *in vivo* 48. Another example comes to aspartate β-hydroxylase (ASPH), a ~86-kDa type II transmembrane protein, belonging to the α-ketoglutarate-dependent dioxygenase family. In HCC tumors, ASPH overexpresses and participates in the malignant transformation process. CRISPR/Cas9-mediated ASPH-knockout (KO) successfully trapped human HCC cells into senescence, thereby retarding HCC progression. It suggests that ASPH can be a potential therapeutic target, which shows a new mechanism that promotes HCC growth by regulating senescence of tumor cells 40 (**Table 2**).

Most recently, by using CRISPR/Cas9-based functional genomics screening of the human kinome (including about 6,000 gRNAs for about 500 different kinases), researchers have found that a set of cyclin-dependent kinases (CDKs), which regulates gene transcription, may be a potential therapeutic target for HCC. Further studies have also indicated that there may be a subgroup of HCC cells with a profound dependence on CDK7 for survival and CDK7 may represent a novel therapeutic target in this subgroup. The high-throughput CRISPR/Cas9 screening technique was first applied to explore the treatment strategy of HCC, providing new approach towards the prevention and treatment of HCC 49. In the future, we will strengthen our exploration in the field of liver and may have the capability to apply the CRISPR/Cas9 technique to HCC.

### HTI

Metabolic liver diseases are better candidates for genome editing correction because many of them are typically severe, refractory to drug therapy and require orthotopic liver transplantation. For some, a low level of gene correction could significantly improve the disease phenotype 50,51. Hereditary tyrosinemia type I (HTI) is a rare autosomal recessive disorder caused by a deficiency of fumarylacetoacetate hydrolase (Fah), the last enzyme that catalyzes the tyrosine catabolic pathway. The mutation of Fah will cause an accumulation of tyrosine and toxic catabolites in the body. The acute form of the disease is characterized by a hepatic failure while the chronic form is characterized by renal dysfunction and neurological crisis, and may lead to death 52. HTI makes for better CRISPR/Cas9 targets because liver cells in which Fah has been repaired have a selective advantage and can expand and repopulate the liver 53.

The potential to correct a Fah mutation mediated by CRISPR/Cas9 has been demonstrated in hepatocytes in a mouse model of HTI. They injected the delivery of Cas9, sgRNA and a coinjected single-stranded DNA(ssDNA) containing the wild-type G nucleotide and homology arms flanking the sgRNA target region by non-viral hydrodynamic injection in the mouse model, which resulted in initial genetic correction rate of ~1/250 cells. The expansion of Fah-positive hepatocytes is sufficient to restore the weight loss of a mouse model of HTI 54. Nevertheless, hydrodynamic injection yielded a low correction rate of 0.4% of hepatocytes. Then a safer and more efficient method of CRISPR delivery was reported. Systemic delivery of Cas9 mRNA by lipid nanoparticles and sgRNA/HDR template by adenovirus or adeno-associated virus (AAV) can correct a Fah mutation in the tyrosinemia mice liver and rescue their body weight loss. In this way, Cas9 nuclease can just express for a short time, making targeted gene editing more effective. The efficiency of correction was >6% of hepatocytes, which is significantly higher than the previous delivery system 55.

A new method called metabolic pathway reprogramming was used to cure HTI mice model successfully. Hydroxyphenylpyruvate dioxygenase (Hpd) is the enzyme that catalyzes the second step of tyrosine catabolism. By deleting Hpd with CRISPR/Cas9 *in vivo*, hepatacytes has been converted from tyrosinaemia type I into the benign tyrosinaemia type III. Then edited hepatocytes will replace the entire liver in only a few weeks. Hpd excision can change tyrosine catabolism, preventing the accumulation of tyrosine and toxic catabolites. Compared with gene therapy, metabolic pathway reprogramming doesn't need to express the wild-type protein of the disease-causing gene continuously and the protein may cause an immune response, limiting long-term expression 51.

It has brought up new ideas about treating HTI and the approach may be suitable for the treatment of a range of metabolic liver diseases. Because of its flexibility and ease in adjusting the target site, CRISPR/Cas9 system has many possibilities in the therapy of metabolic liver diseases.

## Regulation of cellular signaling with CRISPR/Cas9 in liver diseases

Recently, novel designer enzymes, such as the CRISPR/Cas9 RNA-guided nuclease system, have provided technologies for developing advanced therapeutic strategies 56.

Researchers attempted to explore the mechanisms of the tumorigenicity suppression conferred by CRISPR/Cas9-mediated disruption of HBsAg in HCC cells. The results have demonstrated that HBsAg-KO in HCC cells can decrease interleukin (IL)-6 production and inhibite signal transducer and activator of transcription 3 (STAT3) signaling, which highlighted the tumorigenic role of HBsAg. It suggests that the IL-6/STAT3 pathway may be implicated in the HBsAg-mediated malignant potential of HBV-associated HCC 56. The previous study has shown that microRNA-3188 (miR-3188) acts as the markedly overexpressed miRNA in HBV-associated HCC but the mechanism of miR-3188 regulation and cancer-related signaling pathways have not been elucidated. Then scientists manipulated miR-3188 expression in human HCC cell lines by the CRISPR/Cas9 systems 57. The results have proved that miR-3188-KO by CRISPR/Cas9 can significantly increase the expression of zinc fingers and homeoboxes protein 2 (ZHX2), which is a direct target of miR-3188 in HCC cells, thus blocking HBV X protein (HBx)-mediated activation of miR-3188 and Notch signaling pathway 57. HBx has been implicated in HBV-related hepatocarcinogenesis and is considered to be oncogenic 58,59. The Notch signaling pathway is expected to become a new target for the biological treatment of HCC. Compared with non-HCC tissues, Notch1 associates with a higher expression level as well as Notch3, Notch4 60, confirming that the HBx-miR-3188-ZHX2-Notch1 signaling pathway plays an important role in the pathogenesis and progression of HBV-related HCC with a family history of HCC. Furthermore, both the expression level and activity of cell division cycle 42 (CDC42) are up-regulated in HBx-expressing HuH-7 cells 61. The analysis of CDC42 expression in 20 human liver samples has shown that HBV-related HCC tissues have a higher CDC42 expression 62. Deficiency of CDC42 by the CRISPR/Cas9 system can significantly reduce the proliferation of HuH-7 cells promoted by HBx and truly down-regulate IQ Motif Containing GTPase Activating Protein 1 (IQGAP1), which by the way is a downstream effector of CDC42. Together, HBx/CDC42/IQGAP1 signaling pathways are downregulated in HuH-7-HBx CDC42 KO cells 61 (**Figure 4**).

## Current advantages and limitations

The treatment of liver diseases has been sophisticated, which requires and calls for new and better technologies. The ability to edit specific DNA sequences is of paramount importance to advance gene therapy for application to liver diseases 3.

The greatest advantage of the CRISPR/Cas9 system is its simplicity and wide applicability in genome manipulations of almost all biological systems tested to date, including cell lines, stem cells, yeasts, worms, insects, rodents, and mammals. Researchers can also mutate amino acids of Cas9 that are critical to DNA catalysis to produce dead Cas9 (dCas9), which still binds DNA but lacks endonuclease activity. When targeting the transcription start site (TSS) of genes, dCas9 can physically block the passage of RNA polymerase, leading to gene silencing 63. Most importantly, this effect is both controllable and reversible.

To the best of our knowledge, the most exciting application of the CRISPR/Cas9 technology is its potential in the treatment of human diseases. There have been a growing number of preclinical trials targeting various human diseases even though it is currently still at its early stage for clinical applications 4. Some corresponding limitations need to be addressed before clinical application of CRISPR/Cas9 for liver diseases can be achieved.

One of the foremost challenges is the off-target activity 4. For example, the double-strand breaks (DSBs) may widely occur when the gRNA and DNA heteroduplex is formed without strict restrictions 4. Due to the formation of DNA DSBs, Cas9 cutting may lead to cytotoxicity while the modification of Cas9 is irreversible. Bradley's team has shown that DNA breaks introduced by single-guide RNA/Cas9 can frequently resolve into deletions extending over many kilobases. Furthermore, lesions distal to the cut site and crossover events have been identified. The observed genomic damage in mitotically active cells caused by CRISPR/Cas9 editing may have pathogenic consequences 64. For instance, a CRISPR/Cas9-system -direct-targeting p53 and Phosphatase and Tensin homolog deleted on chromosome ten (PTEN) in combination have been constructed and delivered by hydrodynamic tail vein injection to the liver of HBV-transgenic (HBV-Tg) mice 65. The p53 is a tumor suppressor gene and more than 50% of all malignant tumors have mutations in the gene. PTEN, also a tumor suppressor gene, is a negative regulator of the phosphatidylinositol-3-kinase (PI3K)/Akt signaling pathway 66. This study has demonstrated that the CRISPR/Cas9 mediated mutations of p53 and PTEN loci in adult mice are sufficient to accelerate HCC development in HBV-Tg mice without treatment of any chemical carcinogen 65. In another experiment, the liver cancer models have been generated in wild-type mice by using the CRISPR/Cas9 system to target P53 and PTEN 66. These researches have raised a serious concern for clinical applications that any off-target activity may cause undesirable consequences, which is not acceptable towards treatments 4. To alleviate these concerns, several methods have been proposed including selecting gRNAs through various bioinformatics tools to use shorter gRNA, developing sensitive detection methods, improving Cas9 enzymes, constructing effective anti-Cas9 inhibitors 67,68, and amending delivery solutions 4,64. In order to solve the off-target problem of Cas9 system and avoid side effects, many research teams try to add a safe and controllable switch to regulate the system, making the work of Cas9 system have spatial-temporal specificity and conditional restriction. Doxycycline-regulated Cas9 expression induction system has been constructed and gene knockout has been achieved in multiple tissues, which enables safe and controllable gene editing *in vivo* 69. Nihongaki Y. et al. have split Cas9 into two inactive fragments and added a magnet protein to each fragment. When being irradiated by blue light, the magnet proteins come together and the separated Cas9 fragments recombine to activate RNA-guided nuclease. Importantly, the process is reversible: when the light is extinguished, the Cas9 nuclease splits again and its activity can be silenced 70. Our team has also developed a similar CRISPR-Cas9-based light-controlled gene expression device that consists of genomic anchor (dCas9-CIB1 fusion protein), transcriptional activator (CRY2-AD fusion protein), sgRNA and reporter/effector gene. In the absence of blue light, the genomic anchor binds guided by the sgRNA to the targeted sequence (gene promoter sequence), while the activator is freely diffused within nucleus. Upon blue light illumination, CRY2 and CIBI combine with each other, recruiting transcriptional ADs to the targeted sequence (promoter) to activate gene transcription 71.

The second obstacle is the PAM restriction. The precision of the CRISPR/Cas9 DSB activity requires the presence of PAM. CRISPR/Cas9s from different bacterial species have been found to have different PAMs with various lengths and nucleotide compositions. Each type of PAM determines the cutting frequencies of the CRISPR/Cas9 for a given genome. None of the PAMs identified so far or even a combination of all of the known PAMs could cover any whole genome sequences, which may restrict the use of CRISPR/Cas9 technology in some cases. The ideal strategy would be to customize a PAM sequence tailored only to the desired target DNA site through alteration of the responsible PAM interacting amino acids, which has been proved possible by the identification of the amino acids responsible for PAM recognition in both SpCas9 and Staphylococcus aureus Cas9 (SaCas9) 4. Most recently, phage-assisted continuous evolution has been used to evolve an expanded PAM SpCas9 variant (xCas9) that can recognize a broad range of PAM sequences including NG, GAA, and GAT. xCas9 not only broadened PAM compatibility but also has much greater DNA specificity than SpCas9 72.

The third difficulty is the variations of efficiency. The efficiency of CRISPR/Cas9 directed DSB activities varies widely depending on the nucleotide compositions and genomic context of the target protospacer DNA sites as well as the sgRNA secondary structure. Additionally, the genome editing efficiency is also affected by non-homologous end joining (NHEJ) and homology-directed repair (HDR) DNA repair mechanisms 4. Studies have demonstrated that the HDR rate is lower than the NHEJ rate in the liver, limiting the therapy of diseases requiring gene editing by HDR 25. Thankfully, the latest research has revealed the Fanconi anemia pathway to make CRISPR/Cas9 work better in almost all cells 73. For liver diseases requiring a high percentage of gene correction such as liver cancer and HBV, it is still unknown whether CRISPR can restore protein levels to a therapeutic threshold so increasing HDR efficiency is an essential task 25. Great efforts have been made to address these impending issues, and the ongoing progress is encouraging, but much more is needed to fully realize the medical potential of CRISPR/Cas9.

Additionally, there are also some limitations such as the specific delivery to intended target cells and the limitation of immunogenicity of gene modifiers and its delivery agent 3. Viral vectors, which have been widely used in other gene therapy applications, may be employed as an efficient delivery mechanism for gene modifiers. Besides, immune stimulation may result from either the gene modifier itself or from the mechanism of delivery. It is important to assess immune activation as it may diminish efficacy following repeat administrations and cause toxicity in either cases. Immune stimulation has significantly hampered gene therapies in the past 3. But surprisingly, the latest research found that bacteriophages are equipped with “anti- CRISPR” molecules. When the number of anti CRISPR bacteriophages exceeds the “critical point”, it can cooperate to overcome CRISPR/Cas immunity 74. This discovery is a key breakthrough and of great significance to the clinical application of gene editing. Although the application of CRISPR/Cas9 is far-reaching, not all liver diseases are currently amenable to this type of treatment. Reversal of certain hepatic disorders, such as alcohol-induced cirrhosis, is not feasible at present 3. But we believe that the rapid pace of technical improvements and the development of new applications will undoubtedly make the CRISPR/Cas9 system an integral part of liver research in the future.

## Future Expectations and Conclusions

Initially, CRISPR/Cas9, the bacterial defense system, had been used by microbiologists to understand bacterial immunity. Over the past five years, however, researchers have turned CRISPR/Cas9 into a powerful tool for biological research. The CRISPR/Cas9 genome editing system has accelerated scientific research. With further attempting to combine CRISPR/Cas9 system and the latest technology such as single-cell sequencing and single base editing, the treatment of liver diseases will be upgraded to a new level.

As a powerful genome-editing tool, the CRISPR/Cas9 system has been quickly developed into a large-scale function-based screening strategy in mammalian cells 75. Researchers established Cas9/sgRNA screens as a powerful tool for systematic genetic analysis in mammalian cells 76. For further research, the CRISPR screening technique can be used to identify the target gene efficiently, while single-cell sequencing can allow us to dig into the single-cell level. As we all know, even in the same kind of tumor, such as HCC, the heterogeneity of the cells in-focus areas of the same patient or among different patients can be very large. In the future, we may be able to combine the single-cell sequencing for cell detection and CRISPR for high-throughput screening of genes to treat liver diseases, which is in line with the idea of “accurate medicine”.

Recent works in mammalian synthetic biology have increased the applicability of synthetic logic circuits for human cancer therapy. In our previous study, we have constructed the modular AND gate circuits based on CRISPR/Cas9 system and validated novel genetic circuits that selectively and robustly mediate gene expression in human cancer cells, providing a safe, controllable and specific intelligent gene-editing system 77. Although there is no precedent for the genetic circuit as a means of improving or treating liver disease currently, our researchers will strive to explore later. It would be of great interest to extend these circuits to clinical research on liver diseases when the challenges for *in vivo* DNA delivery are overcome (**Figure 5**).

Currently, the safest and most effective biological vector for DNA delivery is AAV. In recent years, AAV-based gene therapy drugs have been approved by the US FDA for pre-clinical trials. The All-in-one AAV-Cas9 system recently developed by our group can effectively regulate lipid metabolism in the liver of mice by targeting the Apao1 gene 78. This provides a potentially useful vector to Cas9-based gene therapy for liver diseases.

To sum up, this review has discussed CRISPR/Cas9 and highlighted its advantages and disadvantages for applications to the treatment of liver diseases. Several studies have already demonstrated that these technologies may be used in a tissue- and patient-specific manner to disable, augment and correct gene function. Ultimately gene modifiers and cell-based therapies will increase the number of disorders that may be permanently corrected and alter how inborn liver diseases and viral hepatic infections are treated. These technologies present a novel, versatile tool for the treatment and cure of many hepatic illnesses. In the future, we even hope to achieve "rehabilitation" of cells, which is the transformation of tumor cells into normal cells through CRISPR/Cas9, and it will be a technology sweeping the world. When humans begin to modify their own source code of life, we know that a new era has come.

## Highlights

- Liver diseases are one of the leading causes of mortality in the world and there is an urgent need for effective and safe treatment.
- CRISPR/Cas9 system has driven progress, improved our understanding of liver diseases and has the potential to revolutionize clinical treatment.
- The applications of CRISPR/Cas9 systems are rapidly expanding and limitations are being overcome.
- CRISPR/Cas9 can be readily applied to make basic science discoveries, and also offers exciting prospects for the treatment of liver diseases.

## Figures and Tables

**Figure 1:** ** The timeline of CRISPR/Cas9.** CRISPR/Cas9: Clustered regularly interspaced short palindromic repeats/CRISPR-associated proteins 9 system; crRNA: CRISPR-derived RNA.

**Figure 2:** ** The structure of type II CRISPR/Cas9 system.** Abbreviations; crRNA: CRISPR-derived RNA; gRNA: guide RNA; tracrRNA: trans-activating crRNA.

**Figure 3:** ** Targets of CRISPR/Cas9 system in liver diseases.** Abbreviations; ASPH: Aspartate β-hydroxylase; cccDNA: covalently closed circular DNA; CXCR4: CXC chemokine receptor 4; eEF2: eukaryotic elongation factor 2; FEN1: Flap structure-specific endonuclease; HbsAg: Hepatitis B surface antigen; NCOA5: Nuclear receptor coactivator 5; NTCP: Sodium-taurocholate co-transporting polypeptide; POLK: Polymerase κ; PTEN: Tensin homolog deleted on chromosome ten; rcDNA: relaxed circular DNA.

**Figure 4:** ** Regulations of CRISPR/Cas9 system in liver diseases.** Abbreviations; CDC42: cell division cycle 42; HBx: HBV X protein; IL-6: interleukin 6; IQGAP1: IQ Motif Containing GTPase Activating Protein 1; MiR-3188: microRNA-3188; STAT3: signal transducer and activator of transcription 3; ZHX2: zinc fingers and homeoboxes protein 2.

**Figure 5:** ** Future expectations of type II CRISPR/Cas9 system.** Abbreviations; CAR-T: chimeric antigen receptor T-cell.

**Table 1:** Applications of CRISPR/Cas9 to viral hepatitis

Species	Target	Cell type	Effect	Function	References (PMID)
hCas9	HBV1.2 S1(3028-3050), P1(1292-1314), PS(261-283; 621-643;648-670), XCp(1742-1764), eE(1876-1898), PCE(2421-2443)	Huh7 cells	Diminish cccDNA and rcDNA production	Inhibit HBV	25137139
pX330-U6-Chimeric_BB-CBh-hSpCas9	HBV1.3 X(1523-1542; 1661-1700; 2338-2357; 2416-2435), ORF X/L	Huh7 and HepG2.2.15 cells	Decrease cccDNA concentration, decrease serum levels of the HBsAg and HBeAg	Inhibit HBV	25843425
SaCas9	HBV ORF S,P	Huh7, hNTCP-HepG2 and HepG2.2.15 cells	Inactivation and preferentially degradation of cccDNA	Inhibit HBV	28785016
SaCas9	HBV Sa1(278-252), Sa3(1862-1889), Sa4(2405-2378)	Huh7, HepG2.2.15 and HepAD38 cells	Decrease HBsAg, HBV DNA and pgRNA levels	Inhibit HBV	29458131
pSpCas9 BB-2A-Puro (PX459)	HBV1.2 ORF S4(368-390), S5 (688-710), XP(1257-1278), CP-BCP(1868-1890), CP-URR(1682-1703)	HepG2.A64 cells	Reduce serum surface-antigen levels	Inhibit HBV	27570484
Cas9n	HBV ORF S1, S2, X1, X2	HeLa, HEK293, HepG2-H1.3, HepG2-H2.2.15, hNTCP-HepG2 cells	Inactivate HBV in chronically and *de novo* infected cells	Inhibit HBV	26334116
Cas9	POLK	Huh7 and HepG2-NTCP cells	Inhibit the conversion of rcDNA into cccDNA, diminish cccDNA formation and the viral infection	Inhibit HBV	27783675
pX330-U6-Chimeric_BB-CBh-hSpCas9	FEN1	Hep38.7-Tet cells, HepG2-hNTCP-C4 cells, Hep38.7-Tet cells, 293FT cells, PXB primary human hepatocytes	Inhibit conversion of rcDNA to cccDNA, reduce cccDNA levels	Inhibit HBV	29928064
FnCas9	HCV RNA	Huh-7.5 cells	Inhibit HCV protein expression	Inhibit HCV	25918406

**Table 2:** Applications of CRISPR/Cas9 to HCC

Species	Target	Cell type	Effect	Function	References (PMID)
Cas9	HBV ORFpreS1/preS2/S	HCC cell lines (PLC/PRF/5, HepG2-2.15, Hep3B, SK-hep1, HLF, and Huh-7) and HEK293F cells	Decrease IL-6 production and inhibit STAT3 signaling	Inhibit HBV-associated HCC	29904948
Cas9	MiR-3188	HepG2 and SMMC7721 cells	Upregulate the expression of ZHX2 and block HBx-mediated activation of Notch signaling	Inhibit HBV-associated HCC	28574502
Cas9	ASPH	Huh7 and HepG2 cells	Guide HCC cells to senescence	Inhibit HCC	26683595
Cas9	eEF2	JHH5 cell lines	Decrease cell proliferation and the growth rate	Inhibit HCC	28060762
Cas9	NCOA5	HCC cell lines (Huh-7, HepG2, Bel-7402, Bel-7404, LM3, SK-Hep-1) and LO2	Suppress EMT	Inhibit HCC	29626478
Cas9	CXCR4	HepG2 cells	Inhibit proliferation, migration and invasion, reverse EMT, increase chemosensitivity, decrease the malignancy	Inhibit HCC	28498420
pSpCas9 BB-2A-Puro (PX459)	G9a	BEL7402, SMMC-7721, THLE-3 cells	Suppress the proliferation and migration, inhibit HCC tumorigenicity	Inhibit HCC	28532996
Dead SpCas9	BAX and BCL2	HepG2 cells	Induce cell apoptosis both *in vitro* and *in vivo*	Inhibit HCC	27595406
Cas9	CDK7	Hep3B and Huh7 cells	Impair proliferation of Hep3B and Huh7 cells	Inhibit HCC	29507396
pSpCas9 BB-2A-GFP (PX458)	p53 and PTEN	Mouse H2.35 cells	Accelerate HCC development	Promote HCC	28584302

## Abbreviations

AAV: adeno-associated virus
AFP: α-fetoprotein
ASPH: aspartate β-hydroxylase
Bax: Bcl2-associated X
Bcl2: B-cell lymphoma 2
cccDNA: covalently closed circular DNA
CDC42: cell division cycle 42
CDKs: cyclin-dependent kinases
CHB: chronic hepatitis B
CRISPR/Cas9: clustered regularly interspaced short palindromic repeats/CRISPR-associated proteins 9
crRNA: CRISPR-derived RNA
CXCR4: CXC chemokine receptor 4
CXCL12: chemokine stromal cell derived factor-1
dCas9: dead Cas9
DSBs: double strand breaks
dsDNA: double stranded DNA
ECM: extracellular matrix
eEF2: eukaryotic elongation factor 2
EMT: epithelial-mesenchymal transition
Fah: fumarylacetoacetate hydrolase
FnCas9: francisella novicida Cas9
H3K9me2: histone H3 lysine 9 di-methylation
HBsAg: hepatitis B surface antigen
HBV: hepatitis B virus
HBV-Tg: HBV-transgenic
HBx: HBV X protein
HCC: hepatocellular carcinoma
HCV: hepatitis C virus
HDR: homology-directed repair
Hpd: hydroxyphenylpyruvate dioxigenase
HTI: hereditary tyrosinemia type I
IL-6: interleukin-6
IQGAP1: IQ motif containing GTPase activating protein 1
KO: knockout
LncRNA: long-chain non-coding RNA
MiR-3188: microRNA-3188
NASH: nonalcoholic steatohepatitis
NCOA5: nuclear receptor coactivator 5
NHEJ: non-homologous end joining
NTCP: sodium taurocholate co-transporting polypeptide
PAM: protospacer-associated motif
pgRNA: pregenome RNA
PI3K: phosphatidylinositol-3-kinase
POLK: polymerase κ
PTEN: phosphatase and tensin homolog deleted on chromosome ten
rcDNA: relaxed circular DNA
REPAIR: RNA editing for programmable A-to-I replacement
RNP: ribonucleoprotein
SaCas9: staphylococcus aureus Cas9
sgRNA: small guide RNA
SpCas9: streptococcus pyogenes Cas9
ssDNA: single strand DNA
STAT3: signal transducer and activator of transcription 3
TALENs: transcription activator-like effector nucleases
tracrRNA: trans-activating crRNA
TSS: transcription start site
ZFNs: zinc finger nucleases
ZHX2: zinc fingers and homeoboxes protein 2
